The article "English Text Recognition Deep Learning Framework to Automatically Identify Fake News" was published in 2022. Journal: Comput Intell Neurosci.

# English Text Recognition Deep Learning Framework to Automatically Identify Fake News

**DOI:** 10.1155/2022/1493493

**Published:** 2022-04-28

**Authors:** Fei Wu, Xiaoyu Luo

**Affiliations:** ^1^Hunan Institute of Engineering, 411104 Xiangtan, Hunan, China; ^2^Hunan University of Technology and Business, 410205 Changsha, Hunan, China

## Abstract

Fake news spreading rapidly worldwide is considered one of the most severe problems of modern technology that needs to be addressed immediately. The remarkable increase in the use of social media as a critical source of information combined with the shaking of trust in traditional media, the high speed of digital news dissemination, and the vast amount of information circulating on the Internet have exacerbated the problem of so-called fake news. The present work proves the importance of detecting fake news by taking advantage of the information derived from friendships between users. Specifically, using an innovative deep temporal convolutional network (DTCN) scheme assisted using the tensor factorization non-negative RESCAL method, we take advantage of class-aware rate tables during and not after the factorization process, producing more accurate representations to detect fake news with exceptionally high reliability. In this way, the need to develop automated methods for detecting false information is demonstrated with the primary aim of protecting readers from misinformation.

## 1. Introduction

Man learns and forms consciousness within the social context. He adopts opinions and constructs a large part of his perceptions based on the data given to him as undisputed knowledge by people he trusts, such as teachers, parents, friends, and information sources. This social transmission of knowledge is at the heart of human civilization. However, often, the information and “knowledge” are wrong, intentionally or not. They are usually written and published to mislead [1], harm an organization, a legal or physical person, or even for economic or political benefits, often using impressive titles, or entirely made to increase readability [2]. Fake news is a yellow press or propaganda done with deliberate misinformation or pranks spread through traditional or social media [3, 4].

Considerable research is being conducted on tactics for combating and suppressing fake news, including disinformation, which is the deliberate distribution of false narratives for political reasons or to undermine social cohesiveness in targeted populations [5]. On the other hand, numerous solutions must be adjusted to individual types of fake news, based, for example, on whether the fake news is actively manufactured or produced inadvertently or unintentionally [6].

The article "English Text Recognition Deep Learning Framework to Automatically Identify Fake News" was published in 2022. Journal: Comput Intell Neurosci.

The difficulty of detecting fake news on social media is mainly because fake news is deliberately written to deceive readers [3, 7]. The content of the information can vary in terms of subject matter and writing style. For example, an actual event may be presented in a misleading context to support something false [8]. As a result, a machine learning model that detects fake news solely through content may not deliver the best results. Instead, we can take advantage of additional information generated by the network, such as the profile of users who interact with the news on social media, to get more accurate results [9].

The problem of detecting fake news [10] on social media has been studied and categorized into three main approaches: content, network, and content - network (hybrid approach) [11]. Content-only strategies focus on analyzing the content of the news (e.g., vocabulary, syntax) and detecting patterns through natural language processing methods. However, to produce satisfactory results, a predefined scope is required, which is difficult to achieve in the case of fake news because of its diversity [12]. Network-based approaches extract information from different networks created by users who interact with the news, such as diffusion or relationship networks. In general, network-based methods perform better in dynamic environments and are more suitable for detecting fake news. Finally, hybrid approaches aim to combine the advantages of content and network-based models, integrating both language features and network information into one model [13].

The overall strategy is to discover awful news through human fact-checking and automated artificial intelligence (machine learning, natural language processing, and network analysis). Research communities have used two fundamental counter-strategies: lowering the importance of fake news and sending out warning messages [10, 14].

In the first strategy, objectionable content is pushed down by the search algorithm, such as the second or later pages of a search engine, making it less likely that visitors will see it (most users scan the first page of search results). However, two issues arise. One is that reality is not always black and white, and fact-checkers frequently differ on classifying the content included in computer training sets, risking false positives, and unjustifiable suppression [15]. Furthermore, because fake news evolves quickly, misleading identifiers may become obsolete in the future.

The second strategy entails attaching warnings to erroneous content by expert fact-checkers. Many studies show that corrections and cautions diminish misperceptions and sharing. Despite some early evidence that fact-checking could backfire, further research has revealed that these backfire effects are infrequent. However, the primary issue is that professional fact-checking is not scalable, i.e., it might take a significant amount of time and effort to research each claim. As a result, many (if not most) bogus claims go unchecked. Furthermore, the process is sluggish, and a warning may miss the peak period of viral propagation. Moreover, signs are usually connected to fake news rather than biased coverage of events.

The article "English Text Recognition Deep Learning Framework to Automatically Identify Fake News" was published in 2022. Journal: Comput Intell Neurosci.

A third strategy prioritizes trustworthy sources such as mainstream media and science communication publications. However, this technique has yielded inconsistent results, as many sites contain hype partisan commentary and confirmation bias, and specific community sections deny all scientific research.

The above, in combination with the fact that users play a key role in how fake news is spread, also users share information with other similar users (friends) and that the characteristics of the network are essential in categorizing or classifying fake news [3], suggesting that the exploring networks of user relationships could greatly facilitate the categorization of fake news [9, 16]. As a result, in this paper, we aim to take advantage of information derived from user friendships and to demonstrate their importance in the problem of detecting fake news. In most cases, standard tensor derivatization or decomposition methods are performed in an unsupervised environment [17]. The class information available for some of the data does not affect them. Instead, our goal is to construct class-aware factor tables using tensor factorization methods. We believe that using class information during and not after the factorization process can give more accurate representations for detecting false news with considerable reliability.

Specifically, using a pioneering DTCN scheme [18] assisted using the tensor Factorization non-negative RESCAL method [19], we can utilize factor-aware tables rather than after the factorization process to produce more accurate representations for localization of fake news with exceptionally high credibility [14].

## 2. Related Literature

Detecting misleading information ([20] p 19) is a constantly evolving problem, and recently, many survey papers have covered the topic of online fake news under numerous different approaches [7, 9].

Zhang and Ghorbani [3] presented a comprehensive overview of the findings relating to fake news. They assessed the harm caused by online fake news by looking at the various components that make up false news, including the source, audience, target, substance, and the broader social environment in which it circulates. The most up-to-date detection technologies are all about detecting the characteristics that signal it when fighting misinformation. Fake news detection was reviewed by comparing existing detection methods and examining existing datasets for supervised training models. Fake news was also classified using pre-existing databases, which the researchers studied. Finally, they outlined several intriguing directions for future research into online fake news.

The article "English Text Recognition Deep Learning Framework to Automatically Identify Fake News" was published in 2022. Journal: Comput Intell Neurosci.

To address the issue of missing ground-truth data, as well as its high dimensionality and possible redundancy, the authors of [21] present a unique unsupervised feature learning technique for extracting discriminative features from the original data. It learns the compressed representation of unlabeled input using recurrent neural network-based asymmetric autoencoders and can elaborate on spectral and spectral-spatial characteristics. Their extractors can be added to the unsupervised segmentation pipeline and followed by any clustering technique. The trials indicated that their techniques produce high-quality segmentation without prior class labels and are one order of magnitude faster than 3-D convolutional AEs. Their methods outperform or perform similarly to previous methodologies, allowing for significant data reduction.

Pérez-Rosas et al. [11] focused on the automatic identification of fake content in online news. While testing their models, the researchers found that their best models could detect false content with the same level of accuracy as humans can. As a result of their work, they offered two datasets to detect fake stories: one based on seven different types of news domains, six different types of news domains, and one that was gathered from the web that included celebrities. They also explained the collection, annotation, and validation method and offered many exploratory analyses to discover counterfeit and authentic news content linguistic variations.

Faustini and Covões [4] suggested a method for detecting false news that relied only on text attributes that could be created independent of the source platform. They tested five datasets, including texts and social media postings, in some language groups and found their findings attractive to baselines. They analyzed the accuracy achieved using a particular set of characteristics to those acquired using other common natural language processing approaches. They then ranked the algorithms in order of highest performance. In terms of the feature set, the bag-of-words technique produced the best results but not being statistically more significant than the other attributes. Finally, they created datasets using various channels, such as websites and social media.

The article "English Text Recognition Deep Learning Framework to Automatically Identify Fake News" was published in 2022. Journal: Comput Intell Neurosci.

Yang et al. [22] developed a text and image information based Convolutional neural network model that could incorporate text and image information with the associated explicit and latent properties. More importantly, it was expandable. They performed trials on a dataset obtained before election procedures and real-world false news records to show that TI-CNN was successful in detecting fake news. The findings demonstrated that using explicit and latent information acquired from multilayer neurons; their method could correctly see bogus info with very high efficiency.

The propagation of fake news has become a global issue, undermining public trust. Fake news and actual news propagate differently on social media. Thus, propagation-based detection systems, which use graph neural networks to form graphs with users as nodes and news sharing chains as edges and simultaneously learn propagation patterns and user preferences, have received much attention. The authors of [23] offer a method for detecting false news using the graph transformer network, which can learn efficient node representations while recognizing functional connections between nodes in the original graph. The proposed method's efficacy is proven by comparison studies utilizing a real-world dataset made of Twitter data.

Antoun et al. [7] proposed techniques for detecting fake news, identifying domains and bots in tweets. They used two distinct approaches to catching fake news. The first used breakthroughs in natural language understanding end-to-end deep learning models to recognize aesthetic distinctions between authentic and counterfeit news pieces. The second was built after the competition and surpassed the winner. The best approach for news domain recognition was a hybrid method that combined named entity characteristics with semantic embeddings generated from end-to-end models [4]. The technique for detecting bots on Twitter consisted of elements taken from news tweets mixed with information from the news tweets. The trials revealed the relevance of several aspects, and the findings suggested that the proposed models performed adequately. They want to enhance false news detection by using elements from fact-checking websites with Google queries.

## 3. Methodology

Sequence modeling problems have been addressed mainly through feedback neural networks. This work proposes to model the situation using TCN, which achieves top performance and reliability. Based on a discrete convergence operator that produces a map of output characteristics by dragging a kernel over the input, the suggested architecture is designed to create a map of output characteristics *f*. Using the multiplication between the kernel and the input stride (i.e., the piece of the input with the same size as the kernel), the output characteristic map is constructed. The depth of the output volume is determined by the number of *M* cores (filters) utilized at each convergent level (i.e., the number of output feature maps). Stride and padding are hyperparameters used to adjust the output feature maps' remaining spatial dimensions [24]. The first can be set to any direction of motion and reflects the distance between two consecutive input strides. Specifically, padding refers to the ability to silently expand the inputs by adding to their limitations (typically zeros) zeros to regulate the size of the output. Without padding, the output dimension would decrease after each convergent level [3, 9, 22].

The article "English Text Recognition Deep Learning Framework to Automatically Identify Fake News" was published in 2022. Journal: Comput Intell Neurosci.

Considering a one-dimensional sequence *x* ∈ R*nT* and a one-dimensional nucleus *w* ∈ R*k*, the *i*-th element of the convergence between *x* and *w* is [18, 22, 25]:

(1) $$\begin{array}{c} f\left(i\right)=\left(x*w\right)\left(i\right)=\sum_{j=0}^{k-1}x\left(i-j\right)w\left(j\right). \end{array}$$

with *f* ∈ R*nT* − *k* + 1 if padding is not used; otherwise, the padding has the dimension of the input, i.e., *f* ∈ R*nT*. The previous equation applies to the case of one-dimensional inputs but can easily be extended to inputs of larger dimensions.

In the model we propose, in addition to the contemporary architecture, we also use a fully probabilistic and self-regression model, which can process arbitrary length sequences and extract a sequence of equal length. The network uses causal (expanded) events to achieve this, and the remaining connections are used to handle substantial historical values. In the proposed TCN, the estimated value at time *t* depends only on previous samples and not on future ones. To achieve this behavior, the causal convergence replaces the standard convergence operator/symbol.

In addition, zero-length padding (filter size ¬ 1) is added to ensure that each level is the same length as the input level. Expanded causal events enhance the network's capabilities further, allowing the network receptive field (i.e., the number of input neurons to which the filter is applied) to increase and its ability to learn long-term dependencies on time series. By this logic, considering a one-dimensional input *x* ∈ R*nT* and a nucleus *w* ∈ R*k*, an expanded convolution output using an expansion factor *d* becomes [4, 22, 26]:

(2) $$\begin{array}{c} f\left(i\right)=\left(x{*}_{d}w\right)\left(i\right)=\sum_{j=0}^{k-1}x\left(i-dj\right)w\left(j\right). \end{array}$$

This is an essential advantage over simple causal convulsions, as in the latter case, the receptive field *r* increases linearly with the lattice depth *r* = *k*(*L* − 1). In contrast, with dilated convulsions, the dependence is exponential *r* = 2*L* − 1*k*, ensuring that the network uses a more extensive history size.

The article "English Text Recognition Deep Learning Framework to Automatically Identify Fake News" was published in 2022. Journal: Comput Intell Neurosci.

Despite the application of expanded convergence, the comprehensive system still needs many levels to learn the dynamics of the inputs. Besides, as it turns out experimentally, the performance often degrades with increasing network depth [27]. The degradation problem was addressed using a deep residual learning framework. Each layer in a typical neural network feeds into the next layer. Each layer in a network with leftover blocks provides the next layer and straight into the levels 2-3 hops away.

There are several interpretations of why residual blocks are lovely and how and why they are one of the essential principles that can enable a neural network to function at a high level on a wide range of tasks. We know, for example, that neural networks are universal function approximators with increasing accuracy as the number of layers grows. However, there is a limit to the number of layers that can be added to improve accuracy. If neural networks were universal function approximators, they should have learned any simplex or complex function. However, because of issues such as vanishing gradients and the curse of dimensionality, it turns out that even with suitably deep networks, it may be unable to learn simple functions such as the identity function. This is unwanted. Furthermore, as the number of layers increases, the accuracy will saturate at some point and subsequently decline. Moreover, in most cases, this is not due to overfitting. As a result, shallower networks can learn faster than deeper networks, which is counterintuitive. However, this is observed in practice and is commonly referred to as the degrading problem. We know that shorter networks outperform deeper equivalents with a few more layers in the degradation problem [19, 21].

In particular, the proposed methodology proposes that for a network of *L* levels with training error *ϵ*, introducing *k* additional levels on it should either leave the error unchanged or improve it. In the worst case, the *k* new added nonlinear levels should learn the identity mapping *y* = *H*(*x*) = *x* where *x* is the output of the *L* level network and *y* is the output of the *L* + *k*-level network. According to the proposed solution, these stacked levels are proposed to fit in a residual mapping *F*(*x*) = *H*(*x*) − *x* instead of the desired *H*(*x*). Thus, the initial mapping is reshaped to *F*(*x*) + *x*, implemented via a simple front-end neural network with shortcut connections. In this way, identity mapping is learned simply by driving stacked level weights to zero values.

The article "English Text Recognition Deep Learning Framework to Automatically Identify Fake News" was published in 2022. Journal: Comput Intell Neurosci.

The architecture used is shown in Figure 1 [18, 22, 28].

At the first level of the network, the information is processed separately from the external data (when available). Later, the individual results will be combined and processed by the deep residual network *L* levels [29]. Each level consists of a residual block with one-dimensional expanded causal convolution, ReLU activation function, and dropout to avoid overfitting [30].

The process in the residual block is as shown in Figure 2 [26, 31, 32].

The output plane consists of a 1 × 1 convolution that allows the network to export a one-dimensional vector *y* ∈ R*nT* with the same dimension as the input vector *x*.

To approach multistep prediction, which essentially means that multidimensional data representation is required, we adopt the RESCAL negative factorization method. RESCAL factorization is a new tensor factorization model that scales very well into large amounts of data and can produce state-of-the-art results in many machine learning problems. More specifically, given an *X* tensor, each slice of *X*_*k*_ is factorized as follows [33, 33, 34]:

(3) $$\begin{array}{c} X_{k}\approx AR_{k}A^{T},\;k=1,\ldots ,m, \end{array}$$

where *A* is an array *n* × *r* containing the latent representations of the *n* entities of the problem and *R*_*k*_ is an array *r* × *r* with the latent interactions of the *r* factors in the *k* dimension of the tensor. Tables *A* and *R*_*k*_ are computed by solving the following minimization problem [30, 35, 36]:

(4) $$\begin{array}{c} \frac{\text{min}}{A,R_{k}}f\left(A,R_{k}\right)+g\left(A,R_{k}\right),\\ f\left(A,R_{k}\right)=\frac{1}{2}\sum_{k}{\left\|X_{k}-AR_{k}A^{T}\right\|}_{f}^{2}, \end{array}$$

is the problem of least squares of factorization and

(5) $$\begin{array}{c} g\left(A,R_{k}\right)=\frac{1}{2}\lambda \left({\left\|A\right\|}_{f}^{2}+\sum_{k}R_{kf}^{2}\right), \end{array}$$

is the normalization term added to avoid overfitting the model.

Relational data such as that generated by social networks can generally be considered non-negative. Therefore, the data in our problem can be factorized using a non-negative version of RESCAL. First, we represent the data using a third-order tensor. Each slice of *T*_*k*_ is factorized as follows:

(6) $$\begin{array}{c} T_{k}\approx AR_{k}A^{T},\;k=1,\ldots ,m, \end{array}$$

where *A* is an array *n* × *r* containing the latent representations of *n* entities and *R*_*k*_ is an array *r* × *r* with the latent interactions of the *r* factors in the *k* dimension of the tensor. Parameters *A* and *R*_*k*_ are calculated by solving the following minimization problem [23, 26, 37]:

(7) $$\begin{array}{c} \frac{\text{min}}{A,R_{k}}f\left(A,R_{k}\right)+g\left(A,R_{k}\right),\\ f\left(A,R_{k}\right)=\sum_{k}{\left\|T_{k}-AR_{k}A^{T}\right\|}_{f}^{2}, \end{array}$$

is the problem of least squares of factorization and

(8) $$\begin{array}{c} g\left(A,R_{k}\right)=\lambda_{A}{\left\|A\right\|}_{f}^{2}+\lambda_{R}\sum_{k}R_{kf}^{2}, \end{array}$$

is the normalization term. The non-negative updates for Tables *A* and *R*_*k*_, respectively, are as follows[38, 39]:

(9) $$\begin{array}{c} A\leftarrow A*\frac{\sum_{k}T_{k}AR_{k}^{T}+T_{k}^{T}AR_{k}}{A\left(\left[\sum_{k}R_{k}A^{T}AR_{k}^{T}+R_{k}^{T}A^{T}AR_{k}\right]+\lambda_{A}I\right.},\\ R_{k}\leftarrow R_{k}*\frac{A^{T}T_{k}A}{A^{T}AR_{k}A^{T}A+\lambda_{R}R_{k}}. \end{array}$$

Figure 3 shows the RESCAL Factorization [40, 41].

The article "English Text Recognition Deep Learning Framework to Automatically Identify Fake News" was published in 2022. Journal: Comput Intell Neurosci.

It is important to note that typically, non-negative tensor factorizations add additional constraints that can lead to complex factor tables that require more time to update, leading to scaling issues.

## 4. Experiments

The model we developed uses the non-negative RESCAL factorization within a TCN. Suppose, we have 2*n* number of news (posts) that have been posted on social media, 2*p* of them with class tags, and the remaining 2(*n* − *p*) without, where *p* < *n*. There is an equal number of false and actual news [42]. First, we create two third-order tensors using binary representation to model user's friendships: *X*_(fake)_ ∈ Ru × *u* × *p* containing all news posts marked as false and *X*_(real)_ ∈ Ru × *u* × *p* with news that has been flagged as valid.

Neighborhood tables represent news posts. By stacking these tables, one after the other, we configure the tensors in a binary way and with whether the user interacted with the fake post - if he is following the user.

It is noted that when we declare that a user has interacted with a post, it means that he has posted the related post/news on his social media profile, in our case, on Twitter. Next, we apply the non-negative RESCAL factorization to the tensors X(fake) and X(real). As a result of the factorization, we end up with tables *A*_fake_ ∈ Ru × *r* and *A*_real_ ∈ Ru × *r*, respectively, through the following non-negative updates that result [39, 43, 44]:

(10) $$\begin{array}{c} A_{\text{fake}}\leftarrow A_{\text{fake}}*\frac{\sum_{k}X_{\left(\text{fake}\right)k}A_{\text{fake}}R_{k}+X_{\left(\text{fake}\right)k}^{T}A_{\text{fake}}R_{k}}{A_{\text{fake}}\left(\left[\sum_{k}R_{k}{\left(A_{\text{fake}}\right)}^{T}A_{\text{fake}}R_{k}^{T}+R_{k}{\left(A_{\text{fake}}\right)}^{T}A_{\text{fake}}R_{k}\right]+\lambda_{A_{\text{fake}}}I\right.}, \end{array}$$

where,

(11) $$\begin{array}{c} R_{k}\leftarrow R_{k}*\frac{\sum_{k}A_{\text{fake}}^{T}X_{\left(\text{fake}\right)k}A_{\text{fake}}}{A_{\text{fake}}^{T}A_{\text{fake}}R_{k}{\left(A_{\text{fake}}\right)}^{T}A_{\text{fake}}+\lambda_{R}R_{k}}, \end{array}$$

(12) $$\begin{array}{c} A_{\text{real}}\leftarrow A_{\text{real}}*\frac{\sum_{k}X_{\left(\text{real}\right)k}A_{\text{real}}R_{k}+X_{\left(\text{real}\right)k}^{T}A_{\text{real}}R_{k}}{A_{\text{real}}\left(\left[\sum_{k}R_{k}{\left(A_{\text{real}}\right)}^{T}A_{\text{real}}R_{k}^{T}+R_{k}{\left(A_{\text{real}}\right)}^{T}A_{\text{real}}R_{k}\right]+\lambda_{A_{\text{real}}I}^{I}\right.}, \end{array}$$

where,

(13) $$\begin{array}{c} R_{k}\leftarrow R_{k}*\frac{\sum_{k}A_{\text{real}}^{T}X_{\left(\text{real}\right)k}A_{\text{real}}}{A_{\text{real}}^{T}A_{\text{real}}R_{k}{\left(A_{\text{real}}\right)}^{T}A_{\text{real}}+\lambda_{R}R_{k}}. \end{array}$$

The posts that were not used in the train set as slices of the tensors belong to the test set and do not have a tag yet. Suppose, we have a set of arrays Μ = {*P*_1_, *P*_2_,…, *P*_2_(*n* − *p*)}, with each array corresponding to a different unlabeled post, where *P*_idx_ ∈ Ru × *u* and idx ∈ [1, 2 (*n* − *p*)]. The *P*_idx_ table is created for each post idx in the known binary way described earlier[45].

The article "English Text Recognition Deep Learning Framework to Automatically Identify Fake News" was published in 2022. Journal: Comput Intell Neurosci.

Next, we perform the non-negative RESCAL factorization on the tensors to generate the new factor tables through the following non-negative updates that occur:

(14) $$\begin{array}{c} A_{\text{fake}}^{\prime }\leftarrow A_{\text{fake}}^{\prime }*\frac{\sum_{k}X_{\left(\text{fake}\right)}^{\prime }A_{\text{fake}}^{\prime }R_{k}+X_{\left(\text{fake}\right)k}^{\prime }A_{\text{fake}}^{\prime }R_{k}}{A_{\text{fake}}^{\prime }\left(\left[\sum_{k}R_{k}A_{\text{fake}}^{TT}A_{\text{fake}}^{\prime }R_{k}^{T}+R_{k}A_{\text{fake}}^{\prime T}A_{\text{fake}}^{\prime }R_{k}\right]+\lambda_{A_{\text{fake}}^{\prime }}^{\prime }I\right.}, \end{array}$$

where,

(15) $$\begin{array}{c} R_{k}\leftarrow R_{k}*\frac{\sum_{k}A_{\text{fake}}^{TT}X_{\left(\text{fake}\right)}^{\prime }A_{\text{fake}}^{\prime }}{A_{\text{fake}}^{TT}A_{\text{fake}}^{\prime }R_{k}A_{\text{fake}}^{TT}A_{\text{fake}}^{\prime }+\lambda_{R}R_{k}}, \end{array}$$

(16) $$\begin{array}{c} A_{\text{real}}^{\prime }\leftarrow A_{\text{real}}^{\prime }*\frac{\sum_{k}X_{\left(\text{real}\right)}^{\prime }A_{\text{real}}^{\prime }R_{k}+X_{\left(\text{real}\right)}^{\prime T}A_{\text{real}}^{\prime }R_{k}}{A_{\text{real}}^{\prime }\left(\left[\sum_{k}R_{k}A_{\text{real}}^{T}A_{\text{real}}^{\prime }R_{k}^{T}+R_{k}A_{\text{real}}^{\prime T}A_{\text{real}}^{\prime }R_{k}\right]+\lambda_{A_{\text{real}}^{\prime }}I\right.}, \end{array}$$

where,:

(17) $$\begin{array}{c} R_{k}\leftarrow R_{k}*\frac{\sum_{k}A_{\text{real}}^{\prime T}X_{{\left(\text{real}\right)}^{k}}A_{\text{real}}^{\prime }}{A_{\text{real}}^{\prime T}A_{\text{real}}^{\prime }R_{k}A_{\text{real}}^{\prime T}A_{\text{real}}^{\prime }+\lambda_{R}R_{k}}. \end{array}$$

Since the Euclidean distance is a known metric for calculating the distance that is regularly used in similar difference calculation problems, we calculate the prediction as follows: Let *l* be the still unknown tag of each post, with *l* ∈ [0, 1], where 0 indicates an authentic post and 1 a false one. Finally, we remove the *P*_idx_ table from *X*′_(fake)_ and *X*′_(real)_, add the next *P*_idx+1_ table from the set of tables *M* to both tensors, and repeat the procedure for the remaining 2(*n* − *p*) posts [46, 47].

The article "English Text Recognition Deep Learning Framework to Automatically Identify Fake News" was published in 2022. Journal: Comput Intell Neurosci.

To evaluate the proposed method, we conducted experiments with two public English-language datasets from two platforms, BuzzFeed and PolitiFact, which include both news content and network information, along with class tags that indicate if each news item is false or true. Content provides information related to the news article's content, such as the title, author, and text, while network information includes information such as user profiles, friendships, and activity. For our evaluation, we use only the knowledge of the network, and in particular, the friendship networks between the users who have posted the relevant news. To reduce the size and sporadicity of the data, we removed the users with node grade <3. Finally, we end up with two tensors of dimensions 182 × 1449 × 1449 and 240 × 1697 × 1697 for the BuzzFeed and PolitiFact datasets, respectively. The Colab environment with GPU was used for the experiments.

To measure the method's performance, we choose the precision evaluation metrics, recall, F1-score, and accuracy, often used in similar problems. The first 70% of the news is the train set, and the remaining 30% is the test set. The number of news items classified as accurate is equal to the number of items marked as false. We perform the experiments ten times, independently for each data set, and record the average results [48, 49].

The results of the process are presented in detail in Table 1.

The abovementioned results show that by using only network data and some class tags, adding class information in the middle and not after the tensor factorization process, and with a small number of factors leading to short computation times, we can achieve outstanding performance, even in problems that require the combination of much heterogeneous information and complex calculations. With this in mind, we can confirm our original hypothesis that explore networks between users that can be helpful in the process of detecting fake news.

The article "English Text Recognition Deep Learning Framework to Automatically Identify Fake News" was published in 2022. Journal: Comput Intell Neurosci.

In conclusion, the use of the proposed method creates a highly efficient TCN which can exploit a sizeable historical size effectively. With this architecture, lower memory requirements are achieved during training, and predictions for later time steps are not made sequentially. Still, they can be calculated in parallel, taking advantage of parameter sharing. In addition, the training of the proposed system is much more stable than that which includes RNNs because it allows avoiding the problem of explosion/disappearance of inclination.

The success of the method is mainly due to the following three reasons [9, 28, 41, 50, 51]:

1. Local connectivity: One set of input neurons is connected to each hidden neuron (according to a specific space-time metric). Compared to a fully linked network, this feature significantly reduces the number of parameters that must be learned and facilitates calculations.
2. Parameter Sharing: The weights used to determine the output neurons in a feature map are the same for each location so that the same kernel is employed. There is less of a learning curve because there are fewer parameters to master.
3. Translation exchange rate: Τhe network is resistant to a possible shift of its input.

## 5. Conclusions

In this work, using an innovative DTCN scheme assisted using the tensor Factorization non-negative RESCAL method, we manage to take advantage of class-aware factor tables rather than after the factorization process to produce more accurate representations in detecting fake news with exceptionally high reliability. Instead of applying factorization and classification separately, we proposed a method that combines them into a standard learning process. This approach uses user friendship networks that have interacted with the news and a set of class tags available for some of the news. We proposed a standard RESCAL negative factorization method to combine this information, which incorporates class tags into the factorization itself. In this way, we successfully arrive at a class-aware tensor-aware semi-supervised derivatization. To evaluate the method, we conducted experiments with two public datasets. The results demonstrate integrating class information into the factorization phase as a single process. They also validated our original hypothesis: how individuals connect with news on social media directly affects the news' legitimacy.

As a future extension, we would like to investigate how the proposed methodology is improved when more information is added to it, both from the network and from the news content. In addition, we plan to evaluate the performance of our approach in more databases and investigate the effect of data size on the scalability of the algorithm. It would be interesting to explore new ways of representing the available information with tensors to integrate it into the proposed method at the methodological level. [52–55].

The article "English Text Recognition Deep Learning Framework to Automatically Identify Fake News" was published in 2022. Journal: Comput Intell Neurosci.

## Figures and Tables

**Figure 1:** Proposed TCN architecture.

**Figure 2:** Residual block.

**Figure 3:** RESCAL factorization.

**Table 1:** Performance of the proposed TCN.

Dataset	Accuracy	Precision	Recall	F1-score
BuzzFeed	93.670	93.770	93.775	93.690
PolitiFact	95.280	95.295	95.290	95.285

## Data Availability

The data used in this study are available from the author upon request.
